The article "The relationship between night shift work and breast cancer incidence: A systematic review and meta-analysis of observational studies" was published in 2022. Journal: Open Med (Wars).

# The relationship between night shift work and breast cancer incidence: A systematic review and meta-analysis of observational studies

**DOI:** 10.1515/med-2022-0470

**Published:** 2022-04-08

**Authors:** Jiaze Hong, Yujing He, Rongrong Fu, Yuexiu Si, Binbin Xu, Jiaxuan Xu, Xiangyuan Li, Feiyan Mao

**Affiliations:** The Second Clinical Medical College, Zhejiang Chinese Medical University, Hangzhou, Zhejiang, China; The First Clinical Medical College, Zhejiang Chinese Medical University, Hangzhou, Zhejiang, China; School of Basic Medical Sciences, Zhejiang Chinese Medical University, Hangzhou, Zhejiang, China; Department of Nutrition, HwaMei Hospital, University of Chinese Academy of Sciences, Ningbo, Zhejiang, China; Department of General Surgery, HwaMei Hospital, University of Chinese Academy of Sciences, Northwest Street 41, Haishu District, Ningbo, 315010, Zhejiang, China

**Keywords:** breast cancer, night shift work, hazard, hormone receptor, menopausal status

## Abstract

The purpose of this study was to investigate the relationship between night shift work and breast cancer (BC) incidence. A search was performed in PubMed, EBSCO, Web of Science, and Cochrane Library databases before June 2021. The exposure factor of this study is night shift work, the primary outcome is the risk of BC. A total of 33 observational studies composed of 4,331,782 participants were included. Night shift work increases the risk of BC in the female population (hazard ratio [HR] = 1.20, 95% confidence interval [Cl] = 1.10–1.31, *p* < 0.001), especially receptor-positive BC, including estrogen receptor (ER)+ BC (HR = 1.35, *p* < 0.001), progesterone receptor (PR)+ BC (HR = 1.30, *p* = 0.003), and human epidermal growth factor receptor 2 (HER2)+ BC (HR = 1.42, *p* < 0.001), but has no effect on HER2− BC (HR = 1.10, *p* = 0.515) and ER−/PR− BC (HR = 0.98, *p* = 0.827). The risk of BC was positively correlated with night shift working duration, frequency, and cumulative times. For women who start night work before menopause, night work will increase the incidence of BC (HR = 1.17, *p* = 0.020), but for women who start night work after menopause, night work does not affect BC (HR = 1.04, *p* = 0.293). Night work can increase the incidence of BC in the female population. The effect of long working hours, frequency, and the cumulative number of night shifts on BC is influenced by menopausal status.

## 1 Introduction

According to the latest study [1], breast cancer (BC) has surpassed lung cancer to become the most commonly occurring cancer in women and the leading cause of cancer death in female patients worldwide [2,3]. Among women, BC accounts for 1/4th among cancer cases and for 1 in 6 cancer deaths [1]. BC occurrence is widely believed to be influenced by both genetics (such as mutations in BRCA) [4,5] and risk factors in the environment [6,7,8]. Therefore, researchers are trying to come up with better prevention strategies for women by adjusting the exposure of BC factors [9,10]. Among all those risk factors, diet and lifestyle are considered to be relatively feasible to be adjusted [11,12]. For example, being sedentary [13], obese [14], smoking [15], eating high-fat and high-sugar foods [16,17] may cause the occurrence of BC.

Long-term night shift work has also been identified as one of the potential risk factors for BC [18,19]. Several occupations are often faced with shifting timetables due to their nature. Some occupations require night shift workers to ensure the 24 h service, such as telecommunications broadcast workers [20], health care workers [21], aviation personnel [22], 24 h on-site service personnel [23], etc. Others need to provide security and maintain order, such as cemetery workers [24] and security personnel [25]. But night shift work is not in accordance with the human circadian rhythm [26]. The circadian rhythm disturbance resulting from the light at night [27] and shift working timetable [28] further leads to undesirable fluctuations in hormone secretion [29], thereby affecting human function [30]. In 2007, “shift work involving circadian disruption” was classified by the International Agency for Research on Cancer (IARC) as a probable cause for female BC (IARC Group 2 A) based on sufficient animal [31] and limited epidemiological evidence [32]. In addition to this, the potential consequences of night shift work, including night eating [33], inverted sleep patterns [34], psychological depression [35], and so forth may also induce BC (occurrence).

Although shreds of evidence have shown that night shift work increases the risk of BC, studies in the past 30 years failed to investigate the clear association between night shift work and BC. Also, studies that have set up the length, frequency, and arrangement parameters of night shifts have shown high inconsistency when it comes to the results. In terms of observational research, a study by Lie et al. [36] demonstrated a significantly increased risk for nurses who worked > 5 years with > 6 consecutive night shifts. However, another study by Sweeney et al. [37] showed that though short-term nocturnal work and night shift work were associated with increased risk of developing BC, the 5-year night time work experience was not associated with a greater possibility of developing BC. Researchers have also reached inconsistent conclusions in many other meta-analyses [38,39]. The purpose of this study is to explore the relationship between night shift work and BC risk through systematic review and meta-analysis of current observational studies.

## 2 Materials and methods

### 2.1 Literature search

In the electronic databases of PubMed, Web of Science, the Cochrane Library, and EBSCO, a comprehensive literature search strategy was performed by retrieving the keywords “breast cancer” and “night-shift work” until June 2021. The complete formula used for retrieval was as follows: (“breast cancer” OR “breast neoplasms” OR “BC”) AND (“circadian disruption” OR “shift work” OR “night work” OR “night” OR “shift” OR “night-shift work” OR “rotating-shift work”). The references of included works of literature were manually reviewed to avoid omitting any potential studies. The population, intervention/exposure, comparison, outcome, and setting (PICOS) criteria were used to aid in the design of the study. This meta-analysis was conducted following the Meta-Analysis of Observational Studies in Epidemiology (MOOSE) guidelines [40]. This meta-analysis’s Prospero registration number was CRD42021270128.

### 2.2 Eligibility criteria and study selection

Specific eligible criteria were formulated as follows: inclusion criteria: (1) The study type falls into the category of observational studies. (2) The main exposure of study was night/shift work, and the outcome was BC risk. (3) The study has available data including hazard ratio (HR) and corresponding 95% confidence interval (CI). (4) The study was published in English. Exclusion criteria: (1) the study had no non-night/shift workers control group. (2) Patients with a previous history of concomitant BC. (3) The study was published in duplicate. (4) The study had no available full text.

Two authors (Jiaze Hong and Yujing He) independently applied a search strategy to select studies from the database and independently reviewed the titles and abstracts of these articles to judge whether they met the inclusion criteria. When in doubt, the full text will be searched for further selection. When necessary, authors are contacted for more information about their research. In case of disagreement, it was discussed with an independent third reviewer (Rongrong Fu). When consensus could not be reached, the study was excluded.

### 2.3 Data extraction

All data were extracted using mutually agreed data collection forms. In order to ensure the objectivity and accuracy of the entered data, two investigators (Yuexiu Si and Binbin Xu) independently extracted data from each study. Disagreements were resolved by consensus by the two investigators or consultation with the third author (Jiaxuan Xu). Information, as follows, was extracted: the author’s name, year of publication, study type, country where the study was performed, age, follow-up time, number of participants, number of BC cases, variables adjusted in the statistical analyses, and outcomes (HR and 95%CI).

### 2.4 Evaluation of quality of the studies

The quality of each included study was evaluated and scored by using the Newcastle-Ottawa Quality Assessment Scale (NOS) checklist, a tool used for quality assessment of non-randomized studies. NOS checklist is classified into three aspects: selection, comparability, and outcome. The maximum score of this checklist is nine, and scores between six and nine were identified to be with higher study quality.

### 2.5 Objectives and endpoints

The primary aim of this study is to evaluate the relationship between night shift work and BC incidence. The secondary objective was to explore the relationship between the incidence of BC and the night shift subgroup, including length of work, frequency of work, cumulative times, age at which night work was initiated, and menopausal status. The adjusted outcomes were uniformly adopted for the processing of relevant data from the included articles.

### 2.6 Statistical analysis

The Stata software version 12 (Stata Corp, College Station, Texas, USA) was used to analyze the data. The CI of HR was set up at 95% to examine the relationship between night shift work and BC risk. To increase the credibility of the results, a random effect model was uniformly adopted in this study. Heterogeneity across included studies was tested by Q statistic and *I* ^2^ statistic to quantitatively evaluate the inconsistency. As for the statistic results, a value of *p* < 0.10 and *I* ^2^ > 50% would be considered to be representative of statistically significant heterogeneity. Sensitivity analysis and publication bias tests were performed to evaluate the stability and reliability of the results when more than ten studies were included. Publication bias was evaluated by the Begg’s rank correlation test and Egger’s linear regression test. *P*-values less than 0.05 were considered to be statistically significant.


**Ethics approval and consent to participate:** Not applicable (this article was provided based on researching in global databases).

## 3 Results

### 3.1 Literature search

Through preliminary search in PubMed, EBSCO, Web of Science, and Cochrane Library databases, a total of 58,425 relevant articles were determined according to the search formula described in Section 2. No other record was identified from other sources. A total of 15,110 duplicate articles were deleted. 12,343 articles were excluded due to the title or abstract. The remaining 972 articles were reviewed through full-text reading. Among them, 939 articles were eliminated resulting from the following reasons: no non-night/shift workers were used as control (*n* = 817); duplicate publication (*n* = 79); no data available for extraction (*n* = 36); and non-English language (*n* = 7). Eventually, 33 articles [20,21,22,24,26,36,37,41,42,43,44,45,46,47,48,49,50,51,52,53,54,55,56,57,58,59,60,61,62,63,64,65,66] consisting of 4,331,782 participants were selected for this meta-analysis. The references of included studies were not included after review. The detailed search and study selection process is shown in Figure 1.

**Figure 1:** A schematic flow for the selection of articles included in this meta-analysis.

### 3.2 Study characteristics

Of the 33 included studies, 10 were cohort studies (4,076,375 participants and 50,686 BC cases), 22 were case-control studies (254,441 participants and 21,807 BC cases), and 1 was a cross-sectional study (966 participants and 56 BC cases). All participants were female. Among the selected studies, 18 studies were conducted in Europe, 7 in North America, 6 in Asia, and 2 in Australia. All studies were published between 1996 and 2021, with follow-up periods ranging from 4.9 to 30 years. Regarding age at recruitment, five studies did not set an upper age limit, and one study did not set a lower age limit. Sixteen studies defined the night shift work. Most studies did not put special requirements forward when it comes to the included participants. There were five studies for the nurse group, one study each in airline compartment attendants, textile workers, telecommunications broadcast workers, military, and electromagnetic field working populations. In addition, the adjustment of potential confounding factors varied in different studies. Common adjustment parameters in the selected studies included age, body mass index (BMI), family history of BC, hormone replacement therapy (HRT), reproductive factors, total energy intake, smoking, alcohol consumption, and physical activity. In order to collect data and evaluate relevant exposure factors, 19 studies required a questionnaire, 9 studies chose interviews, and 5 studies combined both. The characteristics of the included studies are shown in Table 1 and Table S1.

**Table 1:** Characteristics of included observational studies in the meta-analysis

Author, year	Country	Age of recruitment (year)	Age of analysis (year)	Follow-up time (year)	No. of cases	No. of participants	Characteristics
Wegrzyn LR, 2017	America	25–55	54.3 ± 7.2	24	9,541	193,075	The nurses’ health studies I and the nurses’ health studies II
Davis S, 2001	America	20–74	59.8 ± 6.4	6	813	1,606	NA
Wang P, 2015	China	22–85	47.6 ± 11.1	5	712	1,454	NA
Yang W, 2019	China	18–74	60.5 ± 8.7	NA	401	802	The Jiujiang breast cancer study
Åkerstedt T, 2015	Sweden	41–60	51.8 ± 4.7	13	463	13,656	The screening across the lifespan twin study
Knutsson A, 2013	Sweden	19–70	38.9 ± 10.4	16.1	94	4,036	The WOLF (work, lipids, and fibrinogen) occupational cohort study
Szkiela M, 2021	Poland	≥35	57.6 ± 3.9	12	494	1,009	NA
Lie JA, 2011	Norway	35–74	54.4 ± 7.7	17	699	1,594	The Norwegian cohort of nurses
Tynes T, 1996	Norway	≥50	53.2 ± 10.8	30	225	77,583	The telecom cohort; the fertility cohort; the female occupational-cancer cohort
Lie JA, 2006	Norway	27–85	58.3 ± 6.4	NA	537	2,680	NA
Gómez-Salgado J, 2021	Spain	25–60	41.2 ± 10.6	NA	56	966	NA
Papantoniou K, 2016	Spain	20–85	58.5 ± 0.3	NA	1,708	3,486	MCC-Spain study
Hansen J, 2012	Denmark	25–75	NA	NA	267	1,302	A cohort of 91,140 female members of the Danish nurses association
Hansen J, 2001	Denmark	30–54	NA	NA	7,035	138,301	NA
Hansen J, 2012	Denmark	16–66	NA	NA	141	692	A cohort of 18,551 female military employees born during 1929–1968
Menegaux F, 2013	France	25–75	56.9 ± 3.1	NA	1,232	2,549	The cell classification and *in-vitro* lifecycle evaluation study
Rabstein S, 2013	Germany	26–74	56.2 ± 8.6	NA	857	1,749	The gene environment interaction and breast cancer study
Grundy A, 2013	Canada	20–80	57.3 ± 10.3	NA	1,134	2,313	NA
Datta K, 2014	India	30–65	55.6 ± 2.6	NA	50	150	NA
Fritschi L, 2013	Australia	18–80	NA	NA	1,205	2,994	The Breast Cancer Employment and Environment Study
Kojo K, 2005	Finland	38–81	49.6 ± 9.4	NA	45	1098	NA
Bustamante-Montes LP, 2019	Mexico	25–65	49.8 ± 11.3	5	101	202	NA
Pronk A, 2010	China	40–70	52.5 ± 9.1	9	717	73,049	The Shanghai women’s health study
Li W, 2015	China	30–80	57.4 ± 10.5	11	1,709	6,489	A cohort of female textile workers in Shanghai
Sweeney MR, 2020	America	35–74	48.3 ± 5.4	13	3,191	48,451	The sister study
O’Leary ES, 2006	America	≤ 75	59.0 ± 8.2	NA	576	1,161	The electromagnetic Fields and breast cancer on Long Island study
Jones ME, 2019	Britain	≥ 16	55.9 ± 5.6	15	2,059	102,869	The generations study cohort
Schwartzbaum J, 2007	Sweden	15–80	46.1 ± 3.5	18	70	1,148,661	NA
Vistisen HT, 2017	Denmark	≥ 18	NA	4.9	1,245	155,540	NA
Harris MA, 2020	Canada	25–74	40.2 ± 10.5	20	30,775	2,051,315	The population-based Canadian census health and environment cohort
Pham TT, 2019	South Korea	≥ 20	NA	10	1,721	3,442	NA
Koppes LL, 2014	Netherlands	15–64	43.2 ± 8.6	13.9	2,531	285,723	The 14 Dutch labor force surveys
Fernandez RC, 2014	Australia	18–80	NA	NA	145	1,785	The breast cancer, employment and environment study

NA: not available.

### 3.3 Total night shift work

Twenty-five studies (568,838 participants) recorded data about BC risk of total night shift work on the female population. Among those, 18 were case-control studies (170,271 participants and 19,212 BC cases), 6 were cohort studies (397,601 participants and 7,769 BC cases), and 1 was a cross-sectional study (966 participants and 56 BC cases). The results showed that night shift work significantly increased the incidence of BC in women compared to those who never or rarely experienced night shifts (HR = 1.20, 95% CI = 1.10–1.31, *p* < 0.001). The heterogeneity in the included studies was significant (*I* ^2^ = 76.3%). The detailed data is displayed in Figure 2.

**Figure 2:** Forest plot describing the association between night shift work and risk of BC.

### 3.4 The duration of night shift work

Twenty-three out of the selected 33 studies discovered the relationship between the length of night shift work and the incidence of BC. In this study, the length of night shift work is divided into three stages based on 10 and 30 years of night shift work. 20 studies (4,078,910 participants and 66,377 BC cases), 17 studies (3,936,466 participants and 57,411 BC cases), and 13 studies (3,813,835 participants and 51,642 BC cases) in the group of participants with a night shift work duration less than 10 years, 11 to 29 years, and more than 30 years have provided the incidence data of BC, respectively. The results showed that a duration of night shift work less than 10 years (HR = 1.09, 95% CI = 1.01–1.18, *p* = 0.032) (*I* ^2^ = 78.9%), between 11 and 29 years (HR = 1.12, 95% CI = 1.01–1.23, *p* = 0.034) (*I* ^2^ = 69.9%), and more than 30 years (HR = 1.18, 95% CI = 1.02–1.36, *p* = 0.024) (*I* ^2^ = 74.4%) will all increase the incidence of BC with a statistical significance. Also, year-round night work will increase the incidence of BC in women. The detailed data is shown in Table 2.

**Table 2:** Effects of night/shift work on breast cancer incidence

Subgroup analysis	No. of studies	No. of cases	No. of participants	HR	95%CI	*p*	Heterogeneity (*I* ^2^) (%)
Night shift duration was 1–10 years	20	66,377	4,078,910	1.09	1.01–1.18	0.032	78.9
Night shift duration was 11–29 years	17	57,411	3,936,466	1.12	1.01–1.23	0.034	69.9
Night shift duration over 30 years	14	51,642	3,813,835	1.18	1.02–1.36	0.024	74.4
Cumulative night shifts exceeding 500	5	3,690	80,278	1.00	0.75–1.34	0.976	46.0
Cumulative night shifts were 500–1000	7	4,445	82,838	1.15	0.83–1.61	0.404	74.1
Cumulative night shifts exceeding 1000	6	4,389	81,872	1.39	0.99–1.95	0.058	70.0
Age at initiation of night shift was less than 20 years old	3	3,633	177,667	0.79	0.54–1.15	0.220	59.1
Age at initiation of night shift was 20–29 years old	5	5,410	182,075	0.97	0.82–1.15	0.728	0
Age at initiation of night shift was 30–39 years old	4	5,354	181,109	1.15	0.96–1.38	0.138	0
Age at onset of night shift work was over 40 years old	2	2,916	104,618	0.85	0.61–1.18	0.320	0
Night shift duration was 1–9 years in the premenopausal population	8	17,004	345,472	1.13	1.02–1.24	0.016	38.7
Night shift for more than 10 years in the premenopausal population	7	16,910	341,436	1.13	0.95–1.36	0.170	42.8
Night shift duration was 1–9 years in the postmenopausal population	8	17,004	345,472	1.03	0.96–1.09	0.426	12.4
Night shift for more than 10 years in the postmenopausal population	7	16,910	341,436	1.19	1.02–1.39	0.026	48.3

HR: hazard ratio; CI: confidence interval.

### 3.5 The frequency of night shift work

A total of 12 studies have provided data on elucidating the relationship between BC night shift work frequency, including 8 case-control studies and 4 cohort studies. This meta-analysis used the frequency of 5 night shifts per week as the boundary and divided the data into two groups: 1–5 times a week (2,525,009 participants and 41,758 BC cases) and more than 5 times a week (2,526,161 participants and 42,316 BC cases). Each group had 11 studies with extractable data. The results showed that when the night shift work frequency was 1–5 times a week, there was no significant effect on elevating the incidence of BC (HR = 1.08, 95% CI = 0.94–1.24, *p* = 0.308) (*I* ^2^ = 78.6%) (Figure 3a), while when the night shift work exceeded 5 times or more within a week, the incidence of BC would increase with a statistically significant difference (HR = 1.50, 95% CI = 1.02–2.20, *p* = 0.037) (*I* ^2^ = 95.0%) (Figure 3b). The results suggested that high-frequency night work is a risk factor to develop BC.

**Figure 3:** Forest plot describing the association between night shift work frequency and risk of BC. (a) 1–5 times per week. (b) More than 5 times a week.

### 3.6 Cumulative times of night shift work

In terms of the cumulative number of night shifts, 7 studies were conducted on the female population. This meta-analysis grouped the data based on the cumulative number of night shifts of 500 and 1000. Through meta-analysis, the results showed that when the cumulative number of night work is less than 500 times (HR = 1.00, *p* = 0.976) (*I* ^2^ = 46.0%) or between 500–1,000 times (HR = 1.15, *p* = 0.404) (*I* ^2^ = 74.1%), there was no effect on the incidence of BC. However, when the number hits 1000, the incidence rate of BC will increase, though the difference was not statistically significant (HR = 1.39, 95% CI = 0.99–1.95, *p* = 0.058) (*I* ^2^ = 70.0%). The detailed data is given in Table 2.

### 3.7 Age at onset of night shift work

Five studies addressed the association of age at initiation of night shift work against the incidence of BC. Data were divided into “younger than 20 years group,” “20–29 years group,” “30–39 years group,” and “older than 40 years group.” The results showed that participants who started night work before age 20 (HR = 0.79, *p* = 0.220), started night work at age 20–29 (HR = 0.97, *p* = 0.728), started night work at age 30–39 (HR = 1.15, *p* = 0.138), or started night work at age 40 (HR = 0.85, *p* = 0.320) had no effect on BC incidence. The detailed data is given in Table 2.

### 3.8 Menopausal status

Six studies have data revealing the relationship between night shift work and the incidence of BC in people of different menopausal statuses. Five of them are case-control studies (11,241 participants and 5,271 BC cases), and one is a cohort study (48,451 participants and 3,191 BC cases). The results showed that the menopausal status of participants when they first experienced night work is related to the incidence of BC. Starting night work before menopause increases the risk of BC in women with statistical significance (HR = 1.17, 95% CI = 1.02–1.3, *p* = 0.020) (*I* ^2^ = 30.1%) (Figure 4a). What is more noteworthy is that when it comes to women who start night work after menopause, there is no noticeable effect on BC incidence (HR = 1.04, 95% CI = 0.97–1.11, *p* = 0.293) (*I* ^2^ = 0%) (Figure 4b). The results suggested that starting night work before menopause will increase the risk of BC in the female population, in other words, a risk factor of BC.

**Figure 4:** Forest plot describing the association between menopausal status at start of night shift work and risk of BC. (a) Night shift work started before menopause. (b) Night shift work started after menopause.

### 3.9 Menopausal status and duration of night shift work

A total of 8 studies explored the effect of different night shift durations on BC incidence in female populations with different menopausal statuses. The data of premenopausal and postmenopausal night shift work was stratified by 10 years of night shift work, of which, eight studies (345,472 participants and 17,004 BC cases) had extractable data for 1–9 years of night shift work and seven studies (341,436 participants and 16,910 BC cases) had extractable data for more than 10 years of night shift work. The results showed that for females who started night shift work before menopause, a 1–9 years of night shift work increased the incidence of BC (HR = 1.13, *p* = 0.016), but there was no fluctuation of BC incidence against a more than 10 years of night shift work experience (HR = 1.13, *p* = 0.170). The result was also true for females who started night shift work after menopause, with no influence by 1–9-year experience (HR = 0.96, *p* = 0.426) but an increase due to a 10-year experience (HR = 1.19, *p* = 0.026). The detailed data is presented in Table 2.

### 3.10 Different types of BC

A total of 7 articles included aimed to discover the relationship between the night shift work and the types of BC. Seven studies (169,586 participants and 8,153 BC cases) classified the type of BC by estrogen receptor (ER), five studies (13,244 participants and 6,507 BC cases) classified according to progesterone receptor (PR), and five studies (166,471 participants and 6,618 BC cases) classified according to human epidermal growth factor receptor 2 (HER2). The results of this meta-analysis showed that night shift work had a statistically significant effect on inducing receptor-positive BC, including ER+ BC (HR = 1.35, 95% CI = 1.19–1.53, *p* < 0.001) (*I* ^2^ = 0%) (Figure 5a), PR+ BC (HR = 1.30, 95% CI = 1.09–1.54, *p* = 0.003) (*I* ^2^ = 33.8%) (Figure 5b), and HER2+ BC (HR = 1.42, 95% CI = 1.17–1.72, *p* < 0.001) (*I* ^2^ = 0%) (Figure 5c). It would increase the incidence of receptor-positive BC in the female population. Whereas for HER2−BC (HR = 1.10, *p* = 0.515) (*I* ^2^ = 79.9%) (Figure 6a) or ER−/PR− BC (HR = 0.98, *p* = 0.827) (*I* ^2^ = 0%) (Figure 6b), night shift work was not an observable risk factor.

**Figure 5:** Forest plot depicting the association between night shift work and risk of receptor positive BC. (a) ER+ BC. (b) ER+ BC. (c) HER2+ BC.

**Figure 6:** Forest plot depicting the association between night shift work and risk of receptor negative BC. (a) HER2− BC. (b) ER−/PR− BC.

### 3.11 Bias risk assessment

The NOS checklist was adopted in this meta-study in order to evaluate the quality of the included observational studies objectively. According to the results of the quality evaluation conducted by the investigators, 9 studies out of 33 were rated 9 points, 16 studies were rated 8 points, 6 studies were rated 7 points, and 2 studies were rated 6 points. All included studies were of high quality based on methodology. The Risk of bias assessments are documented in Table S2.

### 3.12 Publication bias and sensitivity analysis

For the subgroup with more than 10 included articles, sensitivity analysis and publication bias test were performed. Publication bias was evaluated by the Begg’s rank correlation and Egger’s linear regression test. In this meta-analysis, Begg’s rank correlation and Egger’s linear regression test indicated no publication bias among included articles regarding the HR (*p* > 0.05). Sensitivity analysis was applied to assess whether the individual study affected the overall results or not. The results illustrated that individual studies had little influence on the final results, and the analysis was relatively stable and credible (Figure S1).

## 4 Discussion

According to data analysis, we found that night shift work is a risk factor for BC. To be more detailed, night shift work can increase the incidence of BC in the female population, especially receptor-positive BCs, including ER+ BC, PR+ BC, and HER2+ BC, but no effect on HER2− and ER−/PR− BC. The risk of BC was positively correlated with night shift working duration, frequency, and cumulative times. There was no relationship between the age at initiation of night shift work and BC risk. Continuous night shift work for 1–10 years, 11–29 years, and more than 30 years increased the incidence of BC. Working more than 5 night shifts per week, and the cumulative number of night shifts exceeding 1,000 will increase the risk of BC, but the latter has not yet reached a statistically significant difference. For women who started night work before menopause, night work (especially 1–9 years) will increase the incidence of BC, but there will be no effect on those who work more than 10 years. For women who start night shift work after menopause, BC incidence will not be affected by night shift work until there is more than 10-year (night shift work) experience.

The mechanism of how night shift work can induce BC is still not thoroughly elucidated. The mainstream among the dominant hypothesis is that circadian rhythm disturbances were caused by night shift work [67,68]. The mechanism by which circadian rhythm disorders may induce and/or promote the growth of malignant tumors is believed to be complex and multi-factorial [69]. Reduction in melatonin-dominated hormone secretion [70,71], which is resulted from the disrupted circadian rhythms, is considered as the most likely mechanism [72,73]. The multi-level changes in the endocrine system caused by circadian rhythm disturbance led to the possibility of carcinogenic of female endocrine-responsive breasts [74,75]. The abnormal fluctuation in endogenous hormone secretion due to circadian rhythm disturbance is a carcinogenic signal to the breast cells in female since they are sensitive to hormonal changes. The reduction in melatonin secretion may also be a trigger on the occurrence, promotion, and progression of tumor [76,77]. Several studies on night shift workgroups have shown that night shift work significantly reduces melatonin levels in plasma and delays the peak time of melatonin production [78,79]. The changes in level and time of melatonin production are carcinogenic. Moreover, related experiments have shown that melatonin can inhibit the development of different types of cancer in both *in vitro* and *in vivo* [80], and synergistically enhance the pharmacological effects of other anti-cancer drugs [81,82,83]. It is a chemical substance that can potentially be used as an adjuvant in chemotherapy in cancer treatment [84,85]. Several clinical studies have shown that although melatonin alone does not have the function of tumor regression, the accompanying prescription of melatonin can improve the efficacy of chemotherapy and radiotherapy with less unfavorable side effects [86,87,88,89,90,91].

When it comes to the cellular level, melatonin can protect cells from DNA damage caused by carcinogens. This is achieved by promoting DNA repair through activating related antioxidant pathways [62,92]. Night shift work-related circadian rhythm disruption reduces the secretion of melatonin, thus weakening the ability to repair DNA, leading to more susceptible cells being vulnerable to be affected by external carcinogens [93,94]. As for molecular level, melatonin can resynchronize the rhythm pattern of gene expression, correct the defects of various circadian genes responsible for cancer development in the expression pattern [95,96], and inhibit tumor signal transduction as well as the metabolic activity of cancer cells [97,98]. The disruption of melatonin signaling caused by night shifts upregulates tumor metabolism and stimulates its growth [99,100].

On the overall level, the reduction in melatonin production is upregulative to the gonadal axis [101,102]. As a response modifier of estrogen and progesterone, especially estradiol, melatonin exerts its anti-estrogen effect by interacting with ER-α [103,104,105] and inhibits the BC cell proliferation induced by estradiol [106,107,108]. At the same time, melatonin can downregulate the synthesis of protein growth factors and expression of proto-oncogenes stimulated by ER [109,110] and HER2, hence inhibiting the development of related BC [110,111,112]. Experimental evidence shows that inhibition of melatonin synthesis enhances the proliferation of ER-positive cell lines and promotes BC in HER-2 transgenic mice [113,114]. According to previous studies, long-term exposure to estrogen or increased cell response to estrogen in female is a noticeable risk factor for BC [114,115]. This may explain why night shift work lifts the risk of receptor-positive BC without any effect on HER2− and ER−/PR− BC. Besides, according to the study of Pham et al., night work has no effect on triple-negative BC [59]. In addition, premenopausal women, who depend more on endogenous estrogen secretion compared with postmenopausal women [18,116] normally have a rapid rate of gonadal axis upregulation in night shift work situations with the aid of active gonadal function, resulting in a high circulating level of estrogen in the body [117]. As mentioned, the overall effects of reduced melatonin on BC may partially explain that night-time work induces BC in women who started night shift work before menopause, whereas it has no effect on women who started night shift work after menopause.

The second supporting mechanism of increased risk of developing BC is that numerous hours of continuous night shift work are related to telomerase shortening [118]. Normal circadian rhythm can help maintain the length of telomerase thus adjusting its activity. Under normal circumstances, telomerase activity is influenced by the circadian rhythm, maintaining the length under the responsibility of telomerase [119,120]. Under the circumstances of night shift work, the circadian rhythm and sleep pattern are disrupted, inducing more error generated in the core circadian rhythm genes which regulate the telomere length and rhythm of activity, and eventually lead to telomere instability and DNA repair disorders [121,122]. Genome instability caused by telomere shortening is widely known as a mechanism of tumor development [118]. Moreover, long-term night work prevents the human body from getting enough rest time. In addition to that, continuous high-frequency night work may also represent a higher risk of human function disruption, making it difficult for the human body to quickly adjust itself into sleep mode and modulate the circadian rhythm [69]. This can explain why high frequency (more than five times a week), long time (perennial), and multiple (over 1,000 times) night shifts increase the incidence of BC.

Recently, a relatively new hypothesis states that the suppression of immune surveillance caused by sleep deprivation at night, obesity induced by leptin secretion disorder, and changes in intestinal microbiota are also associated with the increased risk of BC. First of all, sleep deprivation changes the function of the immune system [72]. In the usual circadian sleep-wake mode, the balance between the Th1 cytokines (e.g., IL-2, IL-12, and interferon γ) which dominate during the day is shifted to the Th2 cytokines (e.g., IL4 and IL-10) which normally dominate during sleep at night [123,124]. This alteration reduces immune surveillance, silences the cellular immune response, and induces abnormal cell division, including tumor cells which may lead to malignant tumor [125,126]. Second, night shift work evokes a decrease in leptin level at night [127,128] as well as an imbalance in energy metabolism [70,129], resulting in night shift workers being more likely to be obese [14,130] and develop the metabolic syndrome [131,132]. Compared with other cancers, BC is more closely related to obesity, and obesity can increase the risk of BC through different mechanisms [133,134]. In addition, the imbalance of microbiota in the composition of the intestinal bacterial population (ecological dysbiosis) can change the level of estrogen in plasma [135,136]. On the one hand, this change is mainly caused by dysregulation of estradiol type bacteria, which have β-glucuronidase activity and favors estrogen in the deconjugated state, increasing the number of free estrogens in vascular circulation, which may potentially lead to BC [137,138,139]. On the other hand, it has been shown that these changes in the gut microbiota stimulate the kynurenine pathway, keeping tryptophan away from the melatonin pathway, reducing vascular circulating melatonin level, thereby increasing the risk of BC in women [138,139].

According to the above new views, we believe that for the women who start night shift work after menopause, 1–9 years of night shift work is too short to result in BC as a carcinogenic factor. When it comes to more than 10 years, the exposure to this carcinogenic factor has accumulated to a certain stage, making the risk of BC significantly greater. First of all, ovarian function declines sharply in women after menopause, together with the great reduction in estrogen secretion, while the number of ERs generally increase with age [140], making cells more sensitive to estrogen, which is an important risk factor for BC. Second, postmenopausal women’s autonomic nervous function will be disturbed, which can lead to abnormal metabolic activity in cells/organs [141]. With long-term night shift work, the metabolic rate will be significantly slower, and obesity is prone to induce BC [142,143]. Finally, postmenopausal females are prone to alteration of the gut microbiota. With long-term night work, the human body will aggravate imbalance by reducing the diversity of the microbiome and increasing the ratio of Firmicutes to Bacteroidetes [144,145,146]. These will lead to changes in estrogen, resulting in increased systemic estrogen level [147], combined with the increase in the number of postmenopausal ERs described in the first reason, which increases the risk of BC [37].

For women who started night shift work before menopause, we believe that the following three points may explain why 1–9 working years increase the risk of BC while there is no effect when it comes to more than 10 years. First of all, studies have shown that women under the age of 45 who are on night shifts from 11–20 years will increase the risk of early menopause by 25% [148]. The disturbance of circadian rhythm can affect ovulation and disrupt the regular menstrual cycle, which will induce ovarian failure and accelerate ovarian circulation. The estrogen in the vascular circulation is drastically reduced, which reduces the risk of exposure [26]. Second, as women age, their sleep patterns gradually turn to morning (wake up and fall asleep earlier), and the total length of sleep becomes shorter [149,150]. Studies have shown that longer sleep time (more than the recommended 7–8 h) increases the risk of BC [64] and people who sleep in the morning chronotype have a lower risk of BC than those who sleep in the evening chronotype [26,151]. Therefore, women’s sleep pattern changes with age and the reduction in duration reduces the risk factors for BC. Last but not least, women who started night shift work before menopause are more adapted to the night shift pattern after long night shift work, which means that their metabolism and the ability to regulate intestinal microbes are more in line with the new biological rhythm of night work or shift work in order to quickly adjust the break and circadian rhythm in sleep mode. In addition, we do not rule out the possibility that “some premenopausal women who work on shifts or short-term night work may switch to the daytime schedule earlier due to difficulty in adapting to the rotation or night time schedule,” thus making the effect on BC paradoxically insignificant after 10 years of night shift work in premenopausal women.

The study accomplished by Wang et al. [152] also performed a subgroup analysis based on discovering the relationship between night shift work frequency with BC. They found that each additional 500 times of night shift work would increase BC development by 13% (RR = 1.13, 95% CI = 1.07–1.21), which is consistent with the results of our study. In addition, 5 of the 10 studies included in this meta-analysis were conducted in nurses whose night shift frequency and duration were more regular, making it easier for them to draw dose-response conclusions (that is, each additional night shift will increase certain BC risks). Dun et al.’s study [153] failed to find any relationship between night work and BC. (OR = 1.00, 95% CI = 0.98–1.03). The possible reason for this inconsistency is that some articles have analyzed the effects of night light and/or sleep interruption on BC in their meta-analysis, resulting in interference in the role of night shift work in BC and making research results less reliable.

Though this meta-analysis has reached a comprehensive and objective conclusion, there are still some potential limitations that need to be considered. First, all risk estimations included in the study used random effect models, but the design of methods, study population, sample size, risk assessment, and related confounding factor adjustments vary between studies, which may reduce the credibility of the conclusions. Second, most studies used questionnaires to assess night shift work, and there were also a few studies that employed interviews or questionnaires combined with interviews, making it inevitable that assessment bias or recall bias will arise during the evaluation of night shift work, especially in case-control studies nested in cohorts, which may have potentially biased our findings. Third, attention needs to be paid to the differences between the definition of night shift work in the included studies. There may be heterogeneity among the definitions based on working hours, working habits, and shift system among the observed population. Finally, not all trials have relevant subgroup data, such as BC type subgroup data, menopausal status subgroup data, and so on.

Despite these limitations, this meta-analysis has its own advantages. First, this research includes a great number of observational studies with more than 4 million participants in Asia, Europe, America, and Australia. The large observation population lifts the reliability and authenticity of the conclusions of this study. Second, the study chose to adjust the relevant data of the largest number of potential confounding factors for statistical analysis to improve the accuracy of the conclusions. Finally, the study grouped abstract data (according to BC type, menopausal status or night work frequency, night work duration, the accumulated number of night work, etc.), and conducted subgroup analysis to comprehensively screen for the possibility of the effect of night shift work on different populations and on different BC types. Overall, this meta-analysis has reached some meaningful conclusions, which may provide new recommendations for the prevention of BC in the female population and for employers to formulate a more reasonable night shift system.

## 5 Conclusion

This meta-analysis found that night shift work increases the risk of BC in women, especially receptor-positive BC subtypes, including ER+ BC, PR+ BC, HER2+ BC, and has no effect on HER2− BC and ER−/PR− BC. The risk of BC was positively correlated with night shift working duration, frequency, and cumulative total times. For women who start night work before menopause, night work will increase the incidence of BC, but for women who start night work after menopause, night work has no effect on BC. However, based on the consideration of related limitations, a large-scale prospective cohort study is still needed to further confirm the research conclusions.

## Abbreviations

BC: breast cancer
BMI: body mass index
CI: confidence interval
ER: estrogen receptor
HER2: human epidermal growth factor receptor 2
HR: hazard ratio
HRT: hormone replacement therapy
IARC: international agency for research on cancer
MOOSE: the meta-analysis of observational studies in epidemiology
NOS: the Newcastle-Ottawa quality assessment scale checklist
PICOS: the population, intervention, comparison, outcome and setting criteria
PR: progesterone receptor
